This article has been retracted.

# Application of Bioinformatics Methods to Identify Key Genes and Functions in Chronic Pelvic Pain

**DOI:** 10.1155/2021/7257405

**Published:** 2021-08-02

**Authors:** Wenchao Sun, Qiji Ju

**Affiliations:** Second Department of Anesthesiology, Ningbo No. 6 Hospital, Ningbo, Zhejiang 315040, China

## Abstract

Neuropathologic pain (NPP) occurs in most patients with chronic pelvic pain (CPP), and the unique physiological characteristics of visceral sensory neurons make the current analgesic effect of CPP patients not optimistic. Therefore, this study explored the possible biological characteristics of key genes in CPP through the bioinformatics method. CPP-related dataset GSE131619 was downloaded from Gene Expression Omnibus to investigate the differentially expressed genes (DEGs) between lumbar dorsal root ganglia (DRG) and sacral DRG, and the functional enrichment analysis was performed. A protein-protein interaction (PPI) network was constructed to search subnet modules of specific biological processes, and then, the genes in the subnet were enriched by single gene set analysis. A CPP mouse model was established, and the expression of key genes were identified by qPCR. The results showed that 127 upregulated DEGs and 103 downregulated DEGs are identified. Functional enrichment analysis showed that most of the genes involved in signal transduction were involved in the pathway of receptor interaction. A subnet module related to neural signal regulation was identified in PPI, including CHRNB4, CHRNA3, and CHRNB2. All three genes were associated with neurological or inflammatory activity and are downregulated in the sacral spinal cord of CPP mice. This study provided three key candidate genes for CPP: CHRNB4, CHRNA3, and CHRNB2, which may be involved in the occurrence and development of CPP, and provided a powerful molecular target for the clinical diagnosis and treatment of CPP.

## 1. Introduction

Chronic pelvic pain (CPP) refers to acyclic pain in the pelvic area lasting more than 3 months, including interstitial cystitis/bladder pain syndrome (IC/BPS) common in women and chronic prostatitis/chronic pelvic pain syndrome (CP/CPPS) specific to men [1, 2]. CPP is commonly seen in endometriosis, chronic prostatitis, irritable bowel syndrome, and many serious psychiatric disorders [2–4]. Unfortunately, pain and injury persist even after additional surgery and/or prolonged medication [4]. This undoubtedly has a disastrous impact on the quality of life of patients, resulting in a serious decrease in productivity, impaired sexual function, and serious psychological and life disorders [4–6]. Unfortunately, CPP has not received due attention like other chronic pain [7], and it is urgent to find out the pain mechanism of CPP to reduce the functional impairment of patients.

Studies have found that when CPP lasts much longer than the expected healing time, it often causes damage to specific organs and develops into the neuropathic pain (NPP) state over time, causing visceral allogeneic pain and hyperalgesia of the bladder and adjacent pelvic organs [8, 9]. In addition, some CPP patients are highly similar to some known neurotic syndromes in their pain state [9]. On the other hand, more than half of CPP patients will develop NPP even if no obvious pathological changes were observed during laparoscopy [10], which leads us to speculate that finding the unique expression pattern of neurons in CPP may reduce unnecessary surgery for patients and facilitate drug selection in clinical practice.

While visceral pain is the source of CPP, visceral sensory neurons are often parallel with somatosensory neurons, and patients' pain cannot be significantly improved if visceral pain fibers are ignored in CPP [9, 11]. Due to its unique physiological and pathological characteristics, visceral pain fibers often have a complex path, leading to poor perception of traditional analgesic drugs and traditional analgesic therapy in CPP patients [9, 11, 12]. The present study analyzed the datasets of the dorsal root ganglion (DRG) of the lumbar segment, which contains only somatosensory neurons, and the DRG of the sacral segment, which contains both somatosensory and visceral sensory neurons, by bioinformatics methods [13], to find the key to the differentially expressed genes for help to improve the understanding of the pathogenesis of the CPP, which provided new molecular targets for the treatment.

## 2. Materials and Methods

### 2.1. Data Acquisition

Lumbosacral dorsal root ganglion of the GSE131619 dataset included L4-5 and L6-S1 DRG of 5 adult male and 7 adult male C57BL/6 mice, as well as 12 cases of lumbar DRG sample, and 12 cases of sacral segment DRG sample were downloaded from Gene Expression Omnibus (https://www.ncbi.nlm.nih.gov/geo/query/acc.cgi).

### 2.2. Screening of Differentially Expressed Genes (DEGs)

R package limma analysis was conducted to screen DGR between samples, filter condition was set as |log2(FC)| > 0.5, *P* < 0.05, and R package ggplot2 was used to map the gene expression.

### 2.3. Function and Pathway Enrichment Analysis of DEGs

Online tool Metascape (https://metascape.org/gp/index.html#/main/step1) [14] of DEGs based on gene ontology (GO) was used to describe the biological process (BP), molecular function (MF), and cellular components (CCs) of DEGs. The pathway enrichment analysis is also conducted according to the Kyoto Encyclopedia of Genes and Genomes (KEGG). Threshold is *P* < 0.01, minimum count is 3, and enrichment factor ˃1.5.

### 2.4. Protein-Protein Interaction (PPI) Network Analysis

The PPI network was constructed based on DEGs using String (https://string-db.org/), Visualization with Cytoscape, and the Molecular Complex (MCODE) plug-in in Cytoscape was used to identify network modules with similar functions in PPI.

### 2.5. Single Gene Set Enrichment Analysis (GSEA)

According to the median expression of key genes as the partition condition, the R package msigdbr was used to match the corresponding species, and the differential enrichment of pathways was performed by using the function gseKEGG in the R package clusterProfiler. The screening conditions were *P* < 0.05 and FDR <25%. Finally, the visualization was performed by using the function gseaplot2 in the R package clusterProfiler.

### 2.6. Experimental Animals and Model Construction

Sixteen C57BL/6 mice (6–8 weeks) were purchased from Beijing Vitong Lihua Experimental Animal Technology Co., Ltd., with half male and half female. A CPP mouse model was built according to the previous study [15], and mice were divided into a CPP group and control group (CON), with 8 mice in each group. Mice in the CPP group were intraperitoneally injected with 0.2 mL of a mixture containing complete Freund's fluid (Beyotime, P2036) and normal saline, while mice in the CON group were injected with the same amount of normal saline. Seven days after the operation, the mice were anesthetized with pentobarbital sodium, and the mice were killed by neck breaking. Spinal cord tissue of the L6-S1 segment was collected and fixed with 4% paraformaldehyde, and frozen sections (7 mm) were made for subsequent experiments. All the procedures in this experiment complied with the National Institutes of Health guidelines for the use and care of laboratory animals [16] and were approved by the Medical Ethics Committee.

### 2.7. RT-qPCR

Total RNA was extracted from tissues using Trizol (Sigma-Aldrich, T9424). The cDNA library was synthesized using the PrimeScript™ One Step RT-PCR Kit (RR055A). PCR amplification was performed on Takara PCR Thermal Cycler Dice™ Touch (TP350). The primer sequence is shown in Table 1. The experimental procedures were strictly used in accordance with the manufacturer's protocol, with GAPDH as the reference gene, and 2^−△△CT^ was used for calculation, △△CT = △CT _experimental group_−△CT _control group_; △CT _experimental group_ = CT _target gene, experimental group_−CT _internal reference gene, experimental group_; and △CT _control group_ = CT _target gene, control group_−CT _internal reference gene, control group_.

### 2.8. Statistical Methods

Experimental data were expressed as mean ± standard deviation. The *T* test and One-way ANOVA were performed by GraphPad Prism 9.0. *P* < 0.05 was considered statistically significant.

## 3. Results

### 3.1. Recognition of DEGs

The expression levels of 12,286 genes in lumbar DRG and sacral DRG were analyzed. The median expression values of all the genes in the samples were in a straight line, and the quality control results were good (Figure 1(a)). The expression pattern cluster analysis of the samples was conducted (Figure 1(b)), of which 127 were upregulated and 103 were downregulated (Figure 1(c)).

### 3.2. GO and KEGG Analysis of DEGs

We conducted GO functional enrichment analysis on 230 DEGs and found 337 BP-, 57 CC-, and 58 MF-related GO terms (Figures 2(a)–2(c)). Most GO terms were related to BP, in which most of the genes were closely related to the regulation of membrane potential, behavior, sensory perception of pain, signal release, etc. KEGG analysis results showed that the most significant enrichment pathways were involved in the conduction of nerve signals, such as ECM-receptor interaction, neuroactive ligand-receptor interaction, and axon guidance (Figure 2(d)).

### 3.3. PPI

According to the String database, the PPI network was constructed (Figure 3), and 41 nodes and 282 edges were identified by consensus. MCODE algorithm was used to identify a protein cluster containing three genes of CHRNB4, CHRNA3, and CHRNB2. The enrichment analysis results showed that this subnet module was related to biological processes such as regulation of membrane potential, behavior, signal release, and regulation of neurotransmitter. The expression of CHRNB4, CHRNA3, and CHRNB2 in normal lumbar DRG was lower than that in sacral DRG (Table 2).

### 3.4. GSEAs of Key Genes

In order to analyze the potential functions of CHRNA3, CHRNB2, and CHRNB4, GSEA was performed on KEGG in the highly expressed samples, and the results showed that these three genes were all related to nerve or inflammatory activity (Figure 4).

### 3.5. Identification of Key Genes

RT-qPCR was used to identify the expression of key genes in the spinal cord tissue of mice at the L6-S1 segment. The results showed that the expression levels of CHRNA3, CHRNB2, and CHRNB4 in the spinal cord tissue of mice in the CPP group were significantly downregulated compared with those in the CON group (*P* < 0.05, Figure 5).

## 4. Discussion

Most of the time, only when pain occurred can we became aware of the presence of viscera and the potential or substantial tissue damage [12]. NPP is often associated with the activation of glial cells and changes in immune signals [17]. Injuries such as inflammation and tissue damage are transmitted to the dorsal horn of the spinal cord, and unlike the harmful signals of somatic structure in a specific spinal cord segment, visceral sensation is often transmitted to synapses at multiple spinal cord segment levels, so visceral pain tended to be diffuse and poorly localized [12, 18]. The viscera can project sensory signals to the dorsal horn of the spinal cord, thereby activating the neural reflex pathway, while peripheral or central sensitization can promote the induction and persistence of chronic pain signals [18, 19]. On the other hand, due to the overlap of the regions regulating visceral pain and psychological stress, when the nerve signal was strong enough, the brain stem or cortical region will provide emotional or conscious regulation, resulting in increased pain perception, hyperalgesia, and an adverse cycle between mental stress and pain state [18, 20–22]. Therefore, patients with visceral pain are vulnerable in psychological and physiological aspects and are easily interfered by the environment, inflammation, nervous system, and other factors [22]. Therefore, it is urgent to explore the molecular mechanism associated with visceral pain, in order to interrupt the neural cascade, relieve pain, and improve the quality of life of patients.

The visceral sensory neurons had unique functional characteristics that are different from those of somatosensory neurons [23, 24], which results in that the efficacy of traditional somatosensory analgesic drugs for CPP patients is not up to expectations [11, 13]. Studies had pointed out that nerve injury will lead to adaptive changes of sensory neurons and corresponding pathways in the central nervous system, resulting in abnormal occurrence of neuron-induced signals and changes in epigenetic regulation of gene expression, leading to increased visceral sensitivity [18, 25]. In this study, we used the dataset created by Smith et al. [13], which suggested DRGs in lumbosacral DRG were caused by differences in visceral sensory neurons in the sacral segment. By reidentifying the unique genes uniquely expressed in visceral sensory neurons, it was helpful to select candidate analgesic targets for patients with CPP [23].

The consensus of this study was that 230 DEGs in lumbar DRG and sacral DRG were identified. GO and KEGG analysis showed that these DRGs were closely related to multiple processes of nerve signaling (regulation of membrane potential, sensory perception of pain, and signal release). It might mediate the synaptic connection between splanchnic sensory neurons by participating in multiple receptor interactions (ECM-receptor interaction, neuroactive ligand-receptor interaction, and atron guidance). MCODE was a unique algorithm used to detect tightly connected regions in the PPI network [26], which was often used to explore subnet modules with specific biological functions, and the genes in the subnet were often considered as key genes [27, 28]. Enrichment analysis showed that the subclusters composed of three genes, CHRNB4, CHRNA3, and CHRNB2, were related to the BP associated with the regulation of membrane potential, signal release, and regulation of neurotransmitter, and these genes were highly expressed in normal sacral segment DRG.

GSEA had now become an indispensable part of high-throughput gene expression data analysis, focusing on gene sets and analyzing their common biological pathways or potential functions [29, 30]. In this study, GSEA results showed that CHRNA3 was enriched in neuroactive ligand-receptor interaction, ECM-receptor interaction, and IL-17 signaling pathway-related pathways, while CHRNB2 and CHRNB4 were related to ferroptosis, the toll-like receptor signaling pathway, the hedgehog signaling pathway, cell cycle, the mTOR signaling pathway, and inflammatory mediator regulation of TRP channels, respectively. Most of these signaling pathways mediate nerve injury and the continuation of NPP by participating in neurotoxicity [31], neural activity [32], inflammatory response [33, 34], hyperalgesia [35], nerve healing [36, 37], microglia polarization [38], and oxidative stress [39].

The nicotine and nicotinic acetylcholine receptors (NAChRs) subtype, by a variety of subunits of combinatorial synthesis channel receptor complexes, its structure, and function in the nervous system of diversity, had been found to enhance the presynaptic neurotransmitter and release and affect the excitability of neurons, and when its function declines, it would cause the nervous system dysfunction [40, 41]. A growing number of studies had found that NACHRs had great potential in the treatment of chronic pain as targets for NPP and inflammation control [42, 43]. In this study, we found that the expression of the three NACHR gene clusters consisting of CHRNB4, CHRNA3, and CHRNB2 decreased in the sacral DRG of the CPP model, which was consistent with the results of previous reports related to nerve injury [44, 45].

## 5. Conclusions

In conclusion, this study found the gene differentially expressed in the visceral sensory neurons of the CPP model, which might be the key to the occurrence of CPP, and provided a new analytical target for the drug therapy of CPP. However, few studies have revealed the contribution of these genes in nerve pain, and further studies are needed to verify this.

## Figures and Tables

**Figure 1:** Identification of differentially expressed genes (DEGs). (a) Fiddle plot and (b) heat plot of the gene expression levels between the samples of lumbar DRG and sacral DRG; (c) volcano map of DEGs in lumbar DRG and sacral DRG. Blue represents the lumbar DRG, and yellow represents the sacral DRG. Orange represents upregulated DEGS, and green represents downregulated DEGS. DRG: dorsal root ganglion.

**Figure 2:** Enrichment analysis results of DEGs. (a) BP, (b) CC, (c) MF, and (d) KEGG enrichment analysis are performed for 230 DEGs. BP: biological process; CC: cell component; MF: molecular function; and KEGG: Kyoto Encyclopedia of Genes and Genomes.

**Figure 3:** Protein-protein interaction network of DEGs. *Note.* The dots in the figure represent the protein members in PPI, and the dots in the upper left corner represent the subnet module with CHRNB4 as the core.

**Figure 4:** Single gene set enrichment analysis of key genes (GSEA). *Note.* (a) GSEA highly expressed by CHRNA3; (b) GSEA highly expressed by CHRNB2; and (c) GSEA highly expressed by CHRNB4.

**Figure 5:** Expression of key genes in CPP mice. *Note.* (a) CHRNA3 is detected by qPCR; (b) CHRNB2; and (c) relative expression level of CHRNB4 in the sacral spinal cord of CPP mice. ^*∗*^*P* < 0.05, ^*∗∗*^*P* < 0.01, and ^*∗∗∗*^*P* < 0.001.

**Table 1:** Primer sequences.

		Sequence (5'-3')	Length	Tm	Location
CHRNA3	Forward	TCCAGTTTGAGGTGTCTATGTCT	23	60.4	182–204
	Reverse	TGGTAGTCAGAGGGTTTCCATTT	23	60.9	308–286

CHRNB2	Forward	ATTACGATGGAATCCCGAAGACT	23	60.9	240–262
	Reverse	TCAAAACGTCCGTCAGCATTT	21	60.8	350–330

CHRNB4	Forward	TGGATGATCTCCTGAACAAAACC	23	60.2	89–111
	Reverse	GTTCTCGCTCATTCACACTGAT	22	60.4	214–193

GAPDH	Forward	AGCTTCGGCACATATTTCATCTG	23	61.0	624–646
	Reverse	CGTTCACTCCCATGACAAACA	21	60.5	712–692

**Table 2:** Difference of expression of key genes in normal lumbar DRG and sacral DRG.

	Log FC	Ave. expression	*t*	*P* value	Adj. *P* value	*B*	Expression
Chrna3	2.804	3.919	11.758	1.53 *e* − 11	8.59 *e* − 08	15.754	Down
Chrnb2	1.498	2.621227581	6.545	8.36 *e* − 07	0.000311285	5.873	Down
Chrnb4	2.570	4.011	11.918	1.16 *e* − 11	8.59 *e* − 08	15.996	Down

*Note.* Lumbar DRG samples are used as the comparison matrix for analysis.

## Data Availability

The data used and/or analyzed during the current study are available from all the authors.
